The article "The Mining Algorithm of Maximum Frequent Itemsets Based on Frequent Pattern Tree" was published in 2022. Journal: Comput Intell Neurosci.

# The Mining Algorithm of Maximum Frequent Itemsets Based on Frequent Pattern Tree

**DOI:** 10.1155/2022/7022168

**Published:** 2022-05-18

**Authors:** Xifeng Mi

**Affiliations:** Jiaozuo Normal College, Jiaozuo 454000, China

## Abstract

In the discipline of data mining, association rule mining is an important study topic that focuses on discovering the relationships between database attributes. The maximum frequent itemset comprises the information of all frequent itemsets, which is one of the important difficulties in mining association rules, and certain data mining applications just need to mine the maximum frequent itemsets. As a result, analyzing the maximum frequent itemset mining technique is practical. Considering this, the research introduces FP-MFIA, a new maximum frequent itemset mining approach based on the FP-tree, which is inspired by the data structure of the frequent pattern tree and the idea that the maximum frequent itemset implies all frequent itemsets. First, the FP-MFIA constructs a one-way FP-tree structure, which only has pointers from the root to the leaves, so that only two scans of the FP-tree are required by the FP-MFIA. On the other hand, it redefines a data storage structure MFI-list for maximum frequent itemsets. It can quickly release unnecessary nodes in the FP-tree after scanning it. In this way, not only the information required by the maximum frequent itemsets can be quickly mined but also the space required for storing the maximum frequent itemsets can be reduced, which greatly improves the mining efficiency. Finally, experiments were conducted to compare the mining efficiency of the novel FP-MFIA algorithm to the IDMFIA and DMFIA algorithms. We can see from the findings that the FP-MFIA algorithm is more efficient than the other two techniques.

## 1. Introduction

The base and core of association rule mining are frequent itemset mining, which is an important study direction in the field of data mining [1, 2]. Many scholars have joined this research field since Agrawal. R et al. published the famous algorithm Apriori in 1994 [3] and have undertaken lots of research on the association rules' problem and achieved promising research results [4–6]. Literature [7–9] carried out some optimization work based on the Apriori algorithm, such as the introduction of hashing method, the idea of division, and random sampling, to make mine rules more efficient. However, none of these algorithms can avoid the inherent defects of the Apriori algorithm, that is, during the mining procedure, a significant number of candidate itemsets are formed, and the database needs to be repeatedly scanned, which seriously affects the efficiency of the algorithms. In response to this problem, Han et al. based on the FP-tree, the literature [10], suggested a method called FP-growth for discovering frequent itemsets. The FP-growth algorithm's execution efficiency is substantially superior to that of the Apriori since it does not form candidate itemsets when searching for frequent itemsets and only needs to scan the database twice. However, if the number of large itemsets is too big, and if the obtained FP-tree has many branches and long branches, a huge number of conditional FP-tree will be constructed in the FP-growth algorithm, which is not only time-consuming but also takes up a lot of storage space. It may lead to the low efficiency of the FP-growth algorithm. Therefore, due to the inherent computational complexity of mining frequent itemsets, the above algorithms are still unsatisfactory for mining frequent itemsets with intensive data. For this reason, scholars have proposed a series of researchers to directly search the maximum frequent itemsets [11–13]. Compared with other association rule mining algorithms, they do not generate numerous frequent itemsets so that it can help decrease the generation of redundant itemsets, so the mining speed is faster. Meanwhile, only the maximum frequent itemsets can meet application needs in some cases. Therefore, an in-depth study of the maximum frequent itemset mining algorithm has important research significance for improving the space utilization and time utilization of the algorithms.

Since it was first proposed in 1998, the research on the maximum frequent itemset has received scholars' great attention. They have performed a lot of work on the maximum frequent itemset [14, 15]. For example, the more classic maximum frequent itemset mining algorithms are Max-Miner [16], DepthProject [17], GenMax [18], MAFIA [19], FP-max [20], and Pincer-Search [21]. What's more is that the well-known maximum frequent itemset mining algorithms also include the algorithm DMFI proposed in literature [22], the algorithm DMFIA proposed in literature [23], and the algorithm IDMFIA used in literature [24]. The Max-Miner was first proposed by Bayardo et al. in 1998. It adopts a breadth-first search strategy and proposes a “look-ahead” pruning strategy. Meanwhile, the dynamic sorting method is used to ensure efficient look-ahead prune, which greatly reduces the traversal time. The DepthProject algorithm adopts a depth-first search strategy and a selective projection method. It represents projected transactions by using horizontal binary bit strings with high compression and counting efficiency. But the problem is that both the preprocessing cost based on binary bit string and the postprocessing cost based on statistical support rate cannot be ignored. The GenMax algorithm proposes to use the local maximum frequent itemsets for superset checking, which reduces the overhead of look-ahead pruning to a certain extent. Later, the literature [19] introduced the MAFIA algorithm, which adopts a depth-first search strategy and uses vertical bitmap and dynamic reordering technology for spatial pruning, which has better performance. Based on FP-growth, the literature [20] utilizes an efficient approach called FP-max for maximum frequent itemset mining. It adopts FP-tree to search frequent itemsets and inserts frequent itemsets into an MFI-tree one by one. But the premise is that there is no superset of the itemset in the MFI-tree, and then, the maximum frequent itemset is finally obtained by traversing the MFI-tree. The Pincer-Search algorithm uses bottom-up and top-down bidirectional search strategies to effectively prune candidate itemsets.

The DMFI algorithm has the same search strategy as the Pincer-Search algorithm. It also uses bottom-up and top-down two-way search strategies. When the database is huge, mining the largest frequent itemset is effective. But like the MAFIA algorithm, repeated scans of the database are inevitable. Therefore, the literature [23] introduced the DMFIA algorithm based on the storage structure of the FP-tree. It makes some improvements based on Max-Miner and compresses the relevant information of frequent itemsets. Only two scans of the FP-tree are required without generating conditional pattern bases, but it needs to generate many maximal frequent item candidates. While the IDMFIA algorithm adopts top-down and bottom-up bidirectional search strategies, it does not make full use of infrequent itemsets for dimensionality reduction so that there are still many useless itemsets in the maximum frequent candidate itemsets.

Analyzing the above research, it is found that since the research history of the maximum frequent itemset mining algorithm is not long, there are still many deficiencies in the efficiency of the algorithms [25, 26]. However, the challenge of mining the maximum frequent items lies in the huge amount of data, and the efficiency of the algorithm is the key. Therefore, it is necessary to develop an efficient algorithm that occupies less memory, operates less, and executes faster. Considering this, the research introduces the FP-MFIA algorithm, a new maximum frequent itemset mining approach based on the FP-tree, which is inspired by the data structure of the frequent pattern tree and the idea that the maximum frequent itemset implies all frequent itemsets. The innovation of the new algorithm is as follows:

1. A one-way FP-tree structure is constructed, which only has pointers from the root to the leaves, so that only two scans of the FP-tree are required by the FP-MFIA. Thereby, it reduces the number of generated maximum frequent item candidate set and times of traversing FP-tree, which greatly improves the space utilization.
2. A new data structure MFI-list is adopted to store the maximum frequent itemsets. After scanning the FP-tree, this structure can immediately release numerous useless nodes during the FP-tree, thereby reducing the space required to store the largest frequent itemsets and improving the mining efficiency, especially for the mining of long-pattern frequent itemsets.
3. Finally, experiments were conducted to compare the mining efficiency of the novel FP-MFIA algorithm to the IDMFIA and DMFIA algorithms. We can see from the findings that the FP-MFIA algorithm is more efficient than the other two techniques.

## 2. Related Concepts and Theories

### 2.1. FP-Tree Data Structure and the Relevant Definitions

Next, we will introduce the data structure FP-tree used in the algorithm FP-MFIA to store dataset information [27]. The FP-tree is a data structure commonly used in frequent itemset mining. However, the classic FP-tree is a compressed storage for the transaction database. When the transaction database is very large, the corresponding constructed FP-tree will also be very large, leading to the algorithm taking up a lot of space. In response to this problem, we optimized the FP-tree in the FP-MFIA algorithm and changed it to a one-way data structure, with only pointers from the root to the leaves. Given a transaction database TD and an itemset *IS* = {*s*_1_, *s*_2_, *s*_3_,…, *s*_*m*_} containing m items, the support sup(*t*) of an itemset t(t⊆IS) in TD can be defined as

(1) $$\begin{array}{c} sup\left(t\right)=\frac{N_{t}}{\left|TD\right|}\times 100\text{\%,} \end{array}$$

where *N*_*t*_ is the number of records in *TD* containing *t*, and |*TD*| is the total number of records in the database. The relationship between the support number count(*t*) of *t* in *TD* and the support degree sup(*t*) is shown in

(2) $$\begin{array}{c} \text{count}\left(t\right)=sup\left(t\right)\times \left|TD\right|, \end{array}$$

If the support of itemset *t* satisfies

(3) $$\begin{array}{c} sup\left(t\right)\geq \min\_\sup. \end{array}$$

then *t* is called frequent itemset.

For item set *t*, if it satisfies

(4) $$\begin{array}{c} \left\{\begin{array}{c} sup\left(t\right)\geq \min\_\sup,\\ sup\left(u\right)<\min\_\sup,u⊃t \end{array}\right). \end{array}$$

then *t* is called the maximum frequent itemset, expressed as MFI.

### 2.2. The Construction Process of FP-Tree

#### 2.2.1. The Structure Definition of FP-Tree

The FP-tree is a tree structure, and each node contains five fields, that is, the project name called node_name, the support count called node_count, the child node chain called node_children, the pointer node-link of the next node in the node chain, and the project prefix called node-pre. In addition, it also needs to have a frequent item header table called the Header table, which contains two fields, the item name called item_name, and the header pointer of the node chain called item-links.

#### 2.2.2. The Construction Process of FP-Tree

The construction process of the FP-tree just scans the transaction database twice: the first time generates frequent 1-itemsets, and the second time constructs the FP-tree. During the process of constructing the FP-tree, each transaction is scanned, the items whose support is greater than the user-defined minimum support threshold are inserted, and they are inserted in descending order of support. When inserting items, you need to use a current pointer to assist the insertion. If the current pointer has no child nodes, the node to be inserted is inserted as its leftmost child node. Otherwise, if the child node of the node pointed to by the current pointer has a node with the same node_name value as the item to be inserted, 1 should be added to its node_count value; otherwise, a new node should be created and it should be inserted into the child chain of the node pointed to by the current pointer. After inserting the node, according to the node_name value of the node, it should be inserted into the corresponding item_links chain in the Header table, and the node_link of the node should be modified at the same time.  Table 1 gives the algorithm description of the new FP-tree.

### 2.3. The Example of Constructing a New FP-Tree

**Example 1 .**

Let Table 2 be the transaction database *D*, and the given minimum support number is 3; then, the corresponding FP-tree is displayed in Figure 1.  Figure 2 is the conditional FP-tree based on the *c* node.

All frequent items can be obtained after scanning the database *D* for the first time, arranged in descending order of support to get the itemset *FI*_*k*_ = {bacde}. Then *D* should be scanned for the second time to make a tree. Figure 1 shows the completed FP-tree.

After the FP-tree is constructed, recursive mining can be performed on it. It should be started with the last item in the Header table, and it should be worked your way up. Taking *c* as an example, its conditional pattern base is {{*b*, *a*:2},{*b*:2},{*a*:2}}. Its conditional FP-tree has two branches, as shown in Figure 2. It produces a pattern set: {{*a*, *c*:4},{*b*, *c*:4},{*b*, *a*, *c*:2}}.

## 3. Maximum Frequent Itemset Mining Algorithm Based on FP-Tree

### 3.1. The Idea of the FP-MFIA Algorithm

Inspired by the data structure of the FP-tree and the idea that the maximum frequent itemset implies all frequent items, the research introduces FP-MFIA, a new maximum frequent itemset mining approach based on FP-tree. The FP-MFIA is mainly optimized from the storage structure of the maximum frequent items. First, as introduced in Section 2.2, the FP-MFIA adopts a one-way FP-tree data structure, which only has pointers from the root to the leaves, so that only two scans of the FP-tree are required by the FP-MFIA. Then, the information required to mine the maximum frequent itemsets is obtained, which significantly optimizes the detection efficiency of the FP-MFIA algorithm. Second, we redefine a data storage structure MFI-list. It can quickly release numerous unnecessary nodes in the FP-tree after scanning it, thereby reducing the space required to store the largest frequent itemsets and improving the mining efficiency, especially for the mining of long-pattern frequent itemsets.

### 3.2. Construction of MFI-List

Analyzing the existing maximum frequent itemset mining algorithms, it can be found that the algorithms spend most of the time detecting whether the obtained itemset is the maximum frequent itemset, resulting in low efficiency. Therefore, to reduce the detection time and optimize the mining efficiency of the algorithm, we redefine a data storage structure of maximum frequent itemsets in the FP-MFIA algorithm, called the MFI-list.

The structure of the MFI-list is defined as follows: assuming that the length of the MFI-list is |*L*_*DF*_|, it is composed of MFI-list nodes and maximum frequent itemset linked list list-MFI. The MFI-list node contains three fields: the item name is denoted as node_name, the maximum length is denoted as length, and the pointer to the corresponding maximum frequent itemset linked list is denoted as first_MFI. The last item of the maximum frequent itemset contained in each node in the maximum frequent itemset linked list pointed to by first_MFI must be node_name. The node_MFI of each node in the maximum frequent itemset linked list list_MFI contains two fields: the maximum frequent itemset bit vector is called MFI_BV, and the pointer to the next node_MFI node is called next_MFI. The definition of the maximum frequent itemset bit vector MFI_BV is as follows: suppose there is a maximum frequent itemset {*i*_1_, *i*_2_,..., *i*_m_}, *i*_1_, *i*_2_,..., *i*_m_ is, respectively, the *x*_1_, *x*_2_,..., *x*_m_ item in *L*_*DF*_. Then, the length of the maximum frequent itemset bit vector MFI_BV is *x*_m_, the value of the *x*_1_, *x*_2_,..., *x*_m_ bit is 1, and the other bits are 0.

The construction process of the MFI-list is as follows: traverse the FP-tree in preorder, initialize the MFI-list, and assign a value to the node_pre of each node. Preorder traverses a path from the root to a leaf node. If the node_pre of the parent node of a node has a value, the node_pre of this node is assigned, and the value is the frequent itemset composed of the union of the node_pre of the parent node and the node_name of this node. If the node_count value of a node is greater than or equal to the minimum support min_sup, and the node_count value of one of its child nodes is less than the minimum support min_sup, or it has no child nodes, the node_pre of this child node is assigned a value, and the value is the frequent itemset consisting of the node_name values of all nodes traversed on the path from the root to this child node. At the same time, the candidate maximum frequent itemset composed of the node_name of all nodes traversed on the path from the root to its parent node is converted into a bit vector; then, it is added to the maximum frequent itemset linked list pointed to by the pointer first_MFI of the *p* node in the MFI-list. Suppose the node_name of the *p* node is the same as the node_name of its parent node, its length is compared with *p*- > length. If it is greater than the existing *p*- > length, the *p*- > length value is updated. If all child nodes of a node have been traversed, the node space is released, and the item_links and node_links pointers are accordingly modified.  Table 3 gives a description of the algorithm for constructing the MFI-list storage structure.

After the MFI-list is initialized, the MFI-list is traversed in reverse order according to the support degree from small to large. Each node is scanned in the MFI-list in turn. If the length value of a node is equal to its number in the *L*_*DF*_, the node should be deleted from the Header table and the corresponding node in the FP-tree should be deleted.

### 3.3. Maximum Frequent Itemset Mining Algorithm FP-MFIA Based on FP-Tree

The FP-MFIA algorithm first uses the properties of the FP-tree to scan the transaction database twice, which greatly improves the detection efficiency. Second, a new maximum frequent item storage structure MFI-list is used to find the maximum frequent itemsets according to the elements obtained in the item Header table. The FP-MFIA algorithm considers the frequent items with the minimum support count, and each cycle performs the following operations: the nodes *nd*_1_, *nd*_2_, ..., *nd*_*h*_ are found, which have the same name as the item to be processed in the FP-tree. First, *nd*_1_- > node-pre, *nd*_2_- > node-pre,...,*nd*_*h*_- > node-pre should be converted into bit vectors. Then, for the bit vector of each node *nd*_*i*_- > node_pre, an “AND” operation should be performed with the bit vector of other *nd*_*j*_- > node-pre (1 ≤ *j*< = *h*, *i* ≠ *j*); then, the result will be *n*_*d*_ (bit vector), as shown in

(5) $$\begin{array}{c} n=nd->node\;\_pre\wedge nd_{j}->node\;\_pre. \end{array}$$

If the number “1” in *nd* is greater than or equal to 2, then the sum of node_count is greater than or equal to *s*, and then, the “AND” operation is performed on *n*_*d*_ and the existing maximum frequent itemsets in the MFI-list node, respectively. If a value other than 0 is obtained, the processing of the next node is performed. If all values are 0, it is added to the MFI-list. Then, the next frequent item should be considered. According to the above introduction, Table 4 gives the maximum frequent itemset mining algorithm FP-MFIA based on FP-tree.

### 3.4. Case Analysis

**Example 2 .**

Let Table 5 be the transaction dataset *D*, then min_sup is 2. The mining results of the FP-MFIA algorithm are shown in Figures 3–5, respectively.

First, the FP-tree corresponding to *D* should be constructed, as can be seen in Figure 3. Then, according to the FP-MFIA algorithm, the maximum frequent itemset MFS is obtained.  Figure 4 shows the MFI-list obtained after traversing the FP-tree in preorder, and Figure 5 shows the simplified FP-tree obtained after traversing the MFI-list.

For frequent item *f*, the node_pre of each node obtained by traversing the FP-tree is *abcdf*, *aef*, and *bef*, respectively, and they can be converted into bit vectors of 111101, 100011, and 010011, with the help of

(6) $$\begin{array}{c} 111101\Lambda 100011=100001, \end{array}$$

(7) $$\begin{array}{c} 111101\Lambda 010011=010001, \end{array}$$

(8) $$\begin{array}{c} 100011\Lambda 010011=000011. \end{array}$$

Then, we can get the frequent itemsets *af*, *bf*, and *ef*. Because there is no corresponding MFI_f_ in the MFI-list, *af*, *bf*, and *ef* can be added to the corresponding MFI-list. For frequent item *e*, since its count value is 1, there is no MFI_e_. The final MFI-list is shown in Figure 6. According to the MFI-list, we can get the maximum frequent itemsets {*a*, *f*}, {*b*, *f*}, {*e*, *f*}, {*a*, *e*}, {*b*, *e*}, and {*a*, *b*, *c*, *d*}.

## 4. Experimental Testing and Analysis

To test the mining effectiveness of the FP-MFIA proposed in this study, we conducted a series of experiments among the FP-MFIA, IDMFIA, and DMFIA algorithms.

### 4.1. Experimental Environment and Experimental Database

The experimental environment of this study is as follows: we use a desktop PC to complete the experiments, and its configuration is as follows: the CPU is Intel(R) Core(TM) i7-9700U, the main frequency is 3.0 GHz, the memory is 8G, the operating system is Windows 10, and the development software is Visual C++ 6.0.

The test dataset selected in this study is derived from the classic datasets Mushroom and Connect in UCI (University of California Irvine).  Table 6 gives the relevant parameters of the selected database.

### 4.2. Algorithm Performance Testing and Analysis

To comprehensively evaluate the mining effectiveness of the FP-MFIA algorithm on different types of datasets, we conducted experiments with different support degrees on the above two databases. First, the execution time of FP_MFIA, DMFIA, and IDMFIA is tested in the condition of high support on the two databases. Second, we, respectively, run the FP_MFIA, DMFIA, and IDMFIA algorithms under the condition of low support. However, since the DMFIA algorithm has less support, its execution time exponentially increases, far exceeding the current maximum range of the coordinate axis. Therefore, in order to obtain a more intuitive experimental comparison chart, we only compare the execution efficiency of the FP-MFIA and IDMFIA algorithms when the support degree is small.

#### 4.2.1. Test Analysis on the Mushroom Database

First, we run the three algorithms FP_MFIA, DMFIA, and IDMFIA on the Mushroom database, and Figures 7 and 8, respectively, exhibit their runtime on the Mushroom database.  Figure 7 illustrates the results of the FP_MFIA, DMFIA, and IDMFIA algorithms on the Mushroom database when the minimum support is large (4 levels: 60%, 55%, 50%, and 45%).  Figure 8 illustrates the results of them on the Mushroom database when the minimum support is small (5 levels: 40%, 35%, 30%, 25%, and 20%).

As shown in Figures 7 and 8, the runtime of the FP-MFIA algorithm in the mushroom database generally is less whether the min_sup is large or the min_sup is small. For the Mushroom database, due to its sparse distribution of frequent itemsets, the FP-MFIA algorithm has a greater advantage for sparsely distributed databases. What's more, we can also see from the figures that when min_sup is large, the efficiency of IDMFIA and FP-MFIA is ideal, and the execution time of DMFIA is the longest. However, when the minimum support is small, the execution efficiency of the FP-MFIA algorithm is significantly superior to that of the IDMFIA.

The three algorithms of FP-MFIA, DMFIA, and IDMFIA all use FP-tree to store transaction datasets. The core principle of the DMFIA algorithm is to scan the dataset only once and use the breadth-first search method to analyze the conditional FP-tree mining. But when there are too many items in the dataset, DMFIA will generate lots of invalid candidate itemsets, which will decrease execution efficiency. Although the IDMFIA algorithm adopts the top-down and bottom-up two-way search strategy, it does not make full use of infrequent itemsets for dimensionality reduction so that there are still many useless itemsets in the maximum frequent candidate itemsets. This will also greatly reduce the operating efficiency to a certain extent. However, because FP-MFIA adopts the one-way FP-tree structure and MFI-list storage structure, only two scans of the FP-tree are required by the FP-MFIA. Moreover, the structure of the MFI-list can quickly release numerous unnecessary nodes in the FP-tree after scanning it. In this way, not only the information required by the maximum frequent itemsets can be quickly mined, but also the space required for storing the maximum frequent itemsets can be reduced, which greatly improves the mining efficiency. Therefore, compared with the two algorithms of IDMFIA and DMFIA, FP-MFIA performs more efficiently.

#### 4.2.2. Test Analysis on the Connect Database

At the same time, we also conducted the same test experiments on the intensive database Connect.  Figure 9 shows the results of the FP_MFIA, IDMFIA, and DMFIA algorithms on the Connect database when the min_sup is large (4 bins: 99%, 98%, 97%, and 96%).  Figure 10 illustrates the results of the FP_MFIA, IDMFIA, and DMFIA algorithms on the Connect database when the min_sup is small (5 levels: 95%, 94%, 93%, 92%, and 91%).

Observing the experimental results of Figures 9 and 10 on the Connect dataset, the same conclusion can be drawn: under different minimum support conditions, the overall running time of the proposed FP-MFI algorithm is less than the IDMFIA and DMFIA algorithms. However, since connect is an intensive database, the execution performance of the FP_MFIA, IDMFIA, and DMFIA algorithms on this database is significantly improved compared to their performance on the Mushroom database. As can be found in Figure 9, the running time of the DMFIA algorithm suddenly increases when the support is at 97%. The reason may be that at this level of support, the frequent items in the item Header table suddenly increase, and the dimension of the largest frequent itemset is small, which causes the DMFIA algorithm to calculate the support number for lots of candidate itemsets.

In summary, through the test experiments on the Mushroom and Connect datasets, we can find that no matter in higher support conditions or the lower support conditions, the execution efficiency of the FP-MFIA is generally superior to that of the IDMFIA and DMFIA algorithms. With the decrease in support, FP-MFIA's time efficiency is obviously better than that of the IDMFIA algorithm. However, the FP-MFIA also has some limitations. For example, the candidate itemsets will become more and more as the scale of data continues to grow, resulting in a longer execution time, which will affect the mining efficiency.

## 5. Conclusions

To improve the mining efficiency of intensive data, the research introduces an FP-MFIA algorithm that can efficiently mine the maximum frequent itemsets to deal with long-pattern frequent itemset excavation. The FP-MFIA is mainly optimized from the storage structure of the maximum frequent items. First, it adopts a one-way FP-tree structure, which only has pointers from the root to the leaves, so that only two scans of the FP-tree are required by the FP-MFIA to obtain the information needed to mine the maximum frequent itemsets. Thereby, it reduces the number of generated maximum frequent item candidate sets and times of traversing the FP-tree, which greatly improves the space utilization. Second, a data storage structure MFI-list of maximum frequent itemsets is redefined. After scanning the FP-tree, it can immediately release numerous useless nodes in the FP-tree, thereby reducing the space required to store the maximum frequent itemsets and improving the mining efficiency, especially for the mining of long-pattern frequent itemsets. Finally, through comparative experiments, it can be concluded that the algorithm FP-MFIA has higher time efficiency than DMFIA and IDMFIA in terms of maximum frequent itemset mining. However, the algorithm FP-MFIA also has some limitations. For example, as the scale of data continues to grow, the number of candidate itemsets also increases, which will consume more running time. Therefore, a further in-depth research is needed.

## Figures and Tables

**Figure 1:** FP-tree constructed from the transactional database.

**Figure 2:** Conditional FP-tree based on (c) node.

**Figure 3:** The FP-tree corresponding to transaction database (D).

**Figure 4:** MFI-list obtained after preorder traversal of FP-tree.

**Figure 5:** Preorder traversal of FP-tree and simplified FP-tree obtained after traversing MFI-list.

**Figure 6:** The final MFI-list obtained.

**Figure 7:** Runtime of FP_MFIA, DMFIA, and IDMFIA algorithms on the Mushroom database (when min_sup is large).

**Figure 8:** Runtime of FP_MFIA, DMFIA, and IDMFIA algorithms on the Mushroom database (when min_sup is small).

**Figure 9:** Runtime of different algorithms on the Connect database (when the min_sup is large).

**Figure 10:** Runtime of different algorithms on the Connect database (when the min_sup is small).

**Table 1:** Pseudocode for constructing new FP-tree.

Algorithm 1: The construction algorithm of new FP-tree.
**Input**: Transaction database *D*, minimum support min_sup. In the process of constructing the FP-tree, the node-pre of each node is null, and the node-pre is assigned after the FP-tree is constructed.
**Output**: FP-tree
**Process**:
Scan database *D* to get frequent 1-itemsets, sort them from large to small according to the support degree, and get the frequent item sequence *FI*_1_;
Create a new FP-tree node, assign the value of the node_name to null, and use it as the root node *T*;
Create FP-tree: call Create function
Function Create()
For each transaction in the database *T*_*i*_ do
{Initialize the current pointer in the FP-tree to point to the root node *T*;
Put the items in the transaction *T*_*i*_ that meet the minimum support count requirement into the queue *Q* in descending order of support count;
For each item in the queue *Q* do
FP-tree. Insert(*I*); //Insert I in the child of the node pointed to by the current pointer (if it exists, its counter will be incremented by 1) and move the current pointer to the node
}
Function Insert (char name)//Insert a node with an item named name into the FP-tree
{if the node pointed to by the current pointer has no child nodes or there is no node whose node_name field is name in the child nodes
Then
{Create a new FP-tree node whose node_name field is name；
current- > node_children = node;
current = = node;//Modify the current pointer to point to the new node
current- > node_link = item_head;
item_head = current;//Add it to the item_name linked list whose item_name value is name in the header table
}
else increase the node_count value of the child node by 1 and modify the current pointer to point to it;
}

**Table 2:** The transaction database.

TID	Items	Frequent items in descending order of support
*T*1	Abe	bae
*T*2	*Bd*	*bd*
*T*3	*Bc*	*bc*
*T*4	*Abd*	bad
*T*5	*Ac*	*ac*
*T*6	*Bc*	*bc*
*T*7	*Ac*	*ac*
*T*8	Abce	bace
*T*9	*Abc*	*bac*

**Table 3:** Pseudocode for constructing MFI-list.

Algorithm 2: Algorithm of constructing MFI-list.
**Input**: FP-tree
**Output**: MFI-list
**Process**:
current = *T*://current points to the current node to be traversed, and its initial value points to the tree root *T*
InitStack(s); //initialize stack *s*
There are untraversed paths in the FP-tree
{while (current- > node_count ≥ min_sup)
{current points to a child node that has not been visited;
Push(*s*,current- > node_name);
}
//When there is no child node or the node_count value of the child node is less than min_sup
*MFI* = {collection of items in stack *s*};
Convert the MFI into the corresponding bit vector and link it to the corresponding maximum frequent itemset linked list
current- > node_pre = *MFI*;
While(current has child nodes in the current path)
{pre = current;
current points to its child node;
current- > node_pre = pre- > node_pre∪current- > node_name;//Take the frequent itemset composed of the union of the node_pre of its parent node and the node_name of the node
}}

**Table 4:** Pseudocode of FP-MFIA.

Algorithm 3: The algorithm of FP-MFIA.
**Input:** The FP-tree of transaction database *D*, the Header table of frequent item, the minimum support count *s*, the frequent item list *L*_*DF*_ in *D*
**Output:** The MFI-list
**Process:**
MFI-list = Ø;
Preorder traversal of the FP-tree to obtain a simplified FP-tree, and initialize the MFI-list at the same time;
Traverse the MFI-list and simplify the FP-tree;
*p* = Header table[| Header table|]; //Analyze each node in the Header table in reverse order, *p* first points to the last node;
while(*p* exists){
*p* = *p*- > item_links; //*p* points to the first node in the FP-tree with the same item name
*q* = *q*- > first_MFI; //*q* points to the MFI-list node with the same item name as *p* in the MFI-list
while (*q* exists)
{According to *p*- > item_links and the node_links of the nodes in the FP-tree, find all the nodes *nd*_1_, *nd*_2_,...,*nd*_*h*_ with the item name *p*- > item_name;
for(*i* = 1; *i* ≤ *h*; *i*++)
for(*j* = 1; *j* ≤ *h*; *j*++)
If(*i* ≠ *j*) then
{Convert *nd*_*i*_- > node_pre, *nd*_*j*_- > node_pre to bit vector;
*nd* = *nd*_*i*_;
*n* = *nd*- > node_pre∧*nd*_*j*_- > node_pre;
if(the number of “1” in *nd* > 1) then
{nd.count = *nd*_*i*_- > node_count + *nd*_*i*_- > node_count;//Calculate the support count for *nd*
*q* = *q*- > first_MFI;
If(nd.count ≥ *s*)
{while(*q*- > next_MFI)
if(*nd* is not a subset of an element in the itemset pointed to by *q*）*q* = *q*- > next_MFI;
else break; }
If(*q*- > next_MFI = = null) *q*- > next_MFI = *nd*; }
}}}}

**Table 5:** Transaction database.

TID	Items
*T*1	abcdep
*T*2	abcdf
*T*3	abcdm
*T*4	abcdi
*T*5	abcdho
*T*6	aef
*T*7	befn
*T*8	ae
*T*9	be
*T*10	ad

**Table 6:** The relevant parameters of the database.

Database	Items	The number of the items	The length of each item
Mushroom	119	8124	23
Connect	129	67557	43

## Data Availability

The labeled dataset used to support the findings of this study is available from the corresponding author upon request.
